RETRACTED

# Effects of Pelvic Floor Muscle Massage on the Pregnancy Outcome of Frozen Embryo Transfer in Patients with Thin Endometrium

**DOI:** 10.1155/2022/2803363

**Published:** 2022-06-29

**Authors:** Longying Shen

**Affiliations:** Kuishan Health Center of Rizhao Economic and Technological Development Zone, China

## Abstract

**Objective:**

To observe the effects of pelvic floor muscle mass on the priority outcome of frozen embryo transfer in patients with thin endometrium.

**Methods:**

The patients who were prepared for freeze-thaw embryo transfer were randomly divided into the study group and control group. Both groups of patients began to take estradiol valerate tablets 3 mg on the third day of menstrual cycle and added progesterone for luteal support after 14 days. Both groups selected high-quality embryos for embryo transfer on the day of embryo transfer. The basic information, embryo transfer, intimal thickness, intimal type, clinical pregnancy rate, and early abortion rate of the two groups were compared.

**Results:**

The intimal thickness of patients in the control group and the study group on the second day of menstruation was (0.49 ± 0.03) and (0.45 ± 0.02) and that before progesterone was (1.17 ± 0.03) and (1.20 ± 0.04), respectively (*P* < 0.05). At the same time, the number of excellent embryos in the study group was significantly higher than that in the control group (*P* < 0.05), but there was no significant difference in the number of transplants between the two groups (*P* > 0.05). The proportion of intimal blood flow of type III + II in the study group was significantly higher than that in the control group (*P* < 0.05). The main adverse pregnancy outcomes of the whole group included biochemical pregnancy, early abortion, and ectopic pregnancy. The incidence of biochemical pregnancy in the control group and the study group was 63.3% (38/60) and 40.0% (24/60), respectively. The incidence of biochemical pregnancy in the control group was significantly higher than that in the study group, but there was no significant difference in the incidence of early abortion and ectopic pregnancy between the two groups (*P* > 0.05).

**Conclusion:**

Pelvic floor muscle massage can improve endometrial thickness and subendometrial blood flow, so as to improve the pregnancy rate of frozen thawed embryo transfer patients.

## 1. Introduction

According to the statistics of the World Health Organization (WHO), 5-15% of couples of gestational age have the problem of infertility [1]. At present, there are nearly 40 million infertility patients in China, and they are increasing at the rate of hundreds of thousands every year, so that infertility has become the third largest disease after tumor and cardiovascular and cerebrovascular diseases [2]. Therefore, this problem has become a worldwide medical and social problem. The main reasons for the increase of infertility include the deterioration of environmental quality, the increase of infectious diseases such as sexually transmitted diseases, and the excessive social psychological pressure. In vitro fertilization embryo transfer (IVF-ET) [3], which appeared at the end of the 21st century, is not only the core part of assisted reproductive technology but also an important way to treat infertile patients in modern medicine, thus bringing fertility hope to the majority of infertile patients. However, the clinical pregnancy rate after embryo transfer (ET) did not reach a satisfactory level (30% ~40%) [4]. For in vitro fertilization embryo transfer patients who have or may have severe ovarian hyperstimulation syndrome, in order to avoid further aggravation of their symptoms, embryos can be frozen and transferred after resuscitation. During embryo transfer [5], it is very difficult to intubate the uterine cavity, wait for the diagnostic results after embryo biopsy, and patients who cannot carry out fresh embryo transfer for other special reasons can reduce the burden of patients and increase the cumulative pregnancy rate through freeze-thaw embryo transfer technology [6]. Therefore, embryo freezing has become one of the conventional technologies of reproductive centers [7, 8]. How to improve the endometrial receptivity of patients with frozen thawed embryo transfer, make it reach the endometrial thickness most suitable for embryo implantation [9], grasp the transfer opportunity, and improve the success rate of frozen thawed embryo transfer is a common problem faced by reproductive centers.

RETRACTED

The center adopts the method of integrated traditional Chinese and Western medicine to improve endometrial receptivity and make it reach the most suitable endometrial thickness for embryo implantation, so as to improve the success rate of freeze-thaw embryo transfer [10]. Chinese acupoint massage has a long history in the diagnosis and treatment of infertility, which is one of the precious heritages of traditional Chinese medicine. Its characteristics are as follows: simple method, low-cost, nontoxic, and side effects. By adjusting the balance of yin and yang, it can adjust and strengthen the function of Zang Fu organs in both directions [11]. Combined with drugs, it can improve the absorption of drugs, enhance the exertion of drug properties, and reduce the possible toxic and side effects of drugs [12]. In this study, the medical massager produced by Shanghai Shengsheng Medical Equipment Co., Ltd. was used for pelvic floor muscle massage instead of traditional massage. The motor was used as the vibration element to massage the human pelvic floor through the massage pad in line with ergonomics. The massager stimulates the pelvic floor muscles through specific vibration frequency and intensity, so that the massage part can dredge the meridians, muscle contraction, accelerate blood circulation, and increase the blood perfusion rate of ovary uterus during embryo implantation, so as to improve the pregnancy rate in IVF-ET and improve the pregnancy outcome [13]. It can be seen that the combination of pelvic floor muscle massage and assisted reproductive technology (Art) is a direction worthy of further research and discussion. Compared with traditional massage, pelvic floor muscle massage instrument is safer, noninvasive, and painless, which is easy for patients to accept. More importantly, it can clearly quantify the stimulation intensity and has high repeatability. In addition to the traditional massage technology and art modern technology, the emergence of pelvic floor muscle massage is more conducive to clinical promotion and scientific research. Besides, pelvic floor muscle massage also provides a broader development space for art technology.

## 2. Method

### 2.1. Case Source

120 patients who failed IVF/ICSI-ET treatment or cancelled fresh embryo transfer and underwent freeze-thaw embryo transfer in the reproductive center of our hospital were collected as the research objects. The patients were randomly divided into 60 cases in the study group and 60 cases in the control group. Fill in the observation form according to the requirements of clinical experiment. Our study was approved by the institutional review board of the hospital, and written informed consent was obtained from each participant. Inclusion criteria were as follows: (1) patients who meet the diagnostic criteria of infertility in western medicine; (2) comply with the indications of IVF-ET specified in the notice of the Ministry of Health on revising the technical specifications, basic standards, and ethical principles related to human assisted reproductive technology and human sperm bank; (3) no history of taking estrogen and progesterone drugs in recent 3 months; (4) those who do not get pregnant by transferring fresh embryos in the egg collection cycle; (5) avoid the occurrence of severe ovarian hyperstimulation syndrome; and (6) fresh cycle endometrium is too thin or endometrial lesions are not suitable for transplantation. Exclusion criteria were as follows: (1) comply with the contraindications of IVF-ET specified in the notice of the Ministry of Health on revising the technical specifications, basic standards, and ethical principles related to human-assisted reproductive technology and human sperm bank; (2) exclude hypertension, hyperthyroidism, and other endocrine diseases. (3) patients over 40 years old or with low ovarian response; (4) patients who cancel the cycle due to embryo quality, sudden diseases, and other factors on the day of transplantation; (5) and patients who are unwilling to participate in the study or do not insist on cooperation.

RETRACTED

### 2.2. Treatment

During the freeze-thaw embryo transfer cycle, both groups began to take orally estradiol valerate 3 mg po bid on the third day of the menstrual cycle. After 14 days of continuous application, progesterone was added, and progesterone capsule 150 mg po bid was given every day, progesterone injection 40 mg im QD. On the day of transplantation, 2000 IU im QOD of chorionic gonadotropin for injection was added, and three of them were used for luteal support. The patients in the observation group received pelvic floor muscle massage for 15-20 minutes every day since their menstruation was clean, and the frequency of use was 50 Hz. The specific operations of pelvic floor muscle massage therapy are as follows: (1) preparation: the patient empties the bladder, and the treatment method is sitting; (2) input power: 40 VA; (3) operating frequency: 3400 rpm; and (4) pulse frequency: 75/min. The patients in the control group were not given pelvic floor muscle massage treatment, and the two groups underwent embryo transfer on the 20th day of menstruation (Figure 1).

### 2.3. Observation Index and Detection Method

Endometrial development in transplantation cycle is as follows: B-ultrasound was used to observe the thickness and type of endometrium in the two groups on the 2nd, 10th, and 17th day of menstrual cycle. The B-ultrasound instrument uses the vaginal probe of Aloka-SSD1700 color ultrasound imaging instrument and sector scanning (probe power 5.0 MHz).

Subendometrial blood flow in the two groups is as follows: the type and resistance of subendometrial blood flow were observed by B-ultrasound on the 10th and 17th days of menstrual cycle. Parameters such as peak systolic velocity (*s*), end diastolic blood velocity (*d*), resistant index, RI = (*S* − *D*)/s, and pulsatility index, pi = (*S* − *D*)/vmean are obtained through the machine's own software. Subendometrial blood flow typing is as follows: the endometrial blood flow typing method first used by Chien and others: type I: endometrial blood flow cannot be detected, type II: only subendometrial blood flow can be detected, and type III: the blood flow in and under the endometrium can be detected.

RETRACTED

### 2.4. In Vitro Culture and Embryo Transfer

After the embryos cultured in vitro meet the transfer conditions, the embryos are transferred under the guidance of abdominal B-ultrasound, and the conventional scheme is adopted for the transfer. After the patient's bladder is moderately filled, take the bladder lithotomy position, understand in detail the uterine position, the angle between the uterine body and the cervix, the length of the cervical tube, and the curvature of the cervix through abdominal ultrasound, measure the longest arc of the sagittal plane of the endometrium (i.e., the distance between the internal opening of the cervix and the endometrium of the uterine fundus) twice, and record the average value of the two. According to the direction and curvature of the cervical tube observed by the uterine exploration records and B-ultrasound, bend the outer tube of the transplantation tube (*k* pets 5000 transplantation tube, a product of cook company) into an appropriate curvature, insert it into the internal opening of the cervix along the endometrium, then place the inner tube in an appropriate position, and place the embryo at the thickest place of the endometrium or the place with the best echo of the endometrium under ultrasound.

### 2.5. Efficacy Criteria

The patients were asked to conduct self-test urine pregnancy test 14 days after transplantation, and the pregnancy outcomes of patients in each group were compared. Biochemical pregnancy is as follows: urine test showed positive reaction of HCG or blood 14 days after transplantation *β* − HCG > 10 IU/L; clinical pregnancy is as follows: 20 days after biochemical pregnancy, pregnancy sac, fetal bud, and fetal heart beat were found in utero under B-ultrasound. Early abortion is as follows: embryo loss occurs within 12 weeks of pregnancy.

### 2.6. Statistical Treatment

There is an SPSS 22.0 software package for statistical analysis. The counting data are expressed in percentage (*n* (%)), and chi square test is used. The measurement data were expressed by mean ± standard error and compared statistically by *t*-test, *P* < 0.05.

## 3. Results

### 3.1. Comparison of Intima and Embryo between the Two Groups

The intimal thickness of the control group and the study group on the second day of menstruation was (0.49 ± 0.03) and (0.45 ± 0.02), respectively. And that intimal thickness of the control group and the study group before progesterone was (1.17 ± 0.03) and (1.20 ± 0.04), respectively. The difference was statistically significant (*P* < 0.05). At the same time, the number of excellent embryos in the study group was significantly higher than that in the control group (*P* < 0.05), but there was no significant difference in the number of transplants between the two groups (*P* > 0.05). See Table 1 and Figure 2.

RETRACTED

### 3.2. Comparison of Subintimal Blood Flow Type and Blood Flow Index between the Two Groups

On the 10th day of menstruation, the intimal blood flow of type III + II in the control group and the study group was 36 cases and 34 cases, respectively, and that of type I was 24 cases and 26 cases, respectively. There was no significant difference (*P* > 0.05). On the 17th day of menstruation, the intimal blood flow of type III + II in the control group and the study group was 37 and 56 cases, respectively, and that of type I was 23 and 4 cases, respectively. The proportion of intimal blood flow of type III + II in the study group was significantly higher than that in the control group (*P* < 0.05). See Table 2.

### 3.3. Comparison of Pregnancy Outcomes between the Two Groups

The main adverse pregnancy outcomes of the whole group included biochemical pregnancy, early abortion, and ectopic pregnancy. The incidence of biochemical pregnancy in the control group and the study group was 63.3% (38/60) and 40.0% (24/60), respectively. The incidence of biochemical pregnancy in the control group was significantly higher than that in the study group. However, there was no significant difference in the incidence of early abortion and ectopic pregnancy between the two groups (*P* > 0.05). See Table 3.

## 4. Discussion

Frozen thawed embryo transfer (FET) is a further treatment measure after the failure of in vitro fertilization (IVF)/intracytoplasmic sperm injection (ICSI). The theoretical basis of frozen embryo storage is that tissue cells can inhibit metabolism and biochemical reaction rate during low-temperature freezing storage, which can make frozen thawed embryos survive. And because it increases the cumulative pregnancy rate [14], reduces the risk of multiple pregnancies in the in vitro fertilization cycle, and reduces the occurrence of moderate and severe ovarian hyperstimulation syndrome (OHSS), at the same time, there are many advantages, such as less cost, relatively simple and easy, and shorter time than the repeated egg retrieval cycle. This has attracted the attention of various reproductive centers, and embryo freezing technology has been carried out. As we all know [15], the key to the success of frozen thawed embryo transfer pregnancy is the synchronization of endometrium and embryo development, because embryo implantation is a process of mutual recognition, mutual accommodation, and interaction between embryo and maternal endometrium [16]. In this process, both embryo and endometrium are in a dynamic process of growth and development, only when the embryo develops to the blastocyst stage. Embryo implantation is allowed only when the endometrium proliferates and differentiates to a receptive state. The synchronization of the two is a necessary condition to ensure the successful implantation of embryos [14]. In FET, too thick or too thin endometrium will affect embryo implantation. How to prepare the endometrium for freeze-thaw embryo transfer is an important topic to be discussed in the field of reproductive medicine. Therefore, the best endometrial preparation scheme is the key to ensure successful implantation. At present, there are many endometrial preparation schemes for freeze-thaw embryo transfer. In our center, endometrial blood flow in natural cycle, hormone replacement cycle, and ovulation induction cycle is often used as one of the influencing factors of endometrial receptivity. At present, the most commonly used blood flow parameters are blood pulsatility index (PI) and resistance index (RI). It is generally believed that high PI and RI reflect the increase of blood flow resistance and the decrease of uterine artery blood flow, poor uterine blood perfusion, and blood supply disorder, which may be one of the reasons for the low pregnancy rate. The study found that before embryo transfer, the uterine artery blood flow PI and RI of patients treated with IVF-ET were measured. It was found that there were significant differences between the pregnant group and nonpregnant group. It was considered that the uterine artery Doppler spectrum was related to the time of endometrial embryo reception, and PI and RI were effective indicators to predict the outcome of IVF-ET. Cheng and others believe that endometrial perfusion index can better reflect endometrial receptivity, so as to guide clinical medication to improve endometrial function and select transplantation time, which will have a far-reaching impact on improving the implantation rate and pregnancy rate of IVF-ET. Therefore, how to improve the distribution of subendometrial blood flow in hormone replacement cycle, reduce blood flow resistance, and improve pregnancy rate is a problem to be solved at present. Based on the principle of simple use, exact curative effect, and economic application, this study applied massage to pelvic floor muscle to improve subendometrial blood flow and improve pregnancy rate.

RETRACTED

The motor is used as the vibration source to massage the pelvic floor of the human body through a massage pad in line with ergonomics. It stimulates the pelvic floor muscles through specific vibration frequency and intensity, so that the massage part can dredge the meridians, contract the muscles, and accelerate the blood circulation. Massage integrates the European concept of pelvic floor rehabilitation with China's traditional medical bioinformatics theory and technology. It is a new and unique method. The stimulation time is set at 15-20 min with a fixed time frequency and intensity. The use of electrical stimulation and biofeedback technology can dredge the meridians and stimulate acupoints, so as to awaken the pelvic floor nerves and muscles, promote the blood circulation in the pelvic cavity, regulate the internal environment, contract the pelvic muscles and ligaments, regulate the function of hypothalamus pituitary gonad axis, and increase the uterine blood flow and subendometrial blood flow. Massage is an early method used in clinical prevention and treatment of pelvic floor muscle injury and atrophy at home and abroad. At present, our center uses it to treat infertility. At present, studies have found that the mechanism of electrical stimulation is as follows: by inducing passive muscle contraction and activating some active molecules, it can promote the increase of the number of muscle cells to a certain extent, induce passive muscle contraction, promote muscle blood circulation, improve venous reflux, prevent the accumulation of harmful metabolites in muscle, and indirectly affect the metabolic process of atrophic muscle cells.

The characteristics of basin massage include the following: ① safe and effective, nontoxic, and side effects. For a safe and effective method, the treatment purpose is achieved through physical methods, which not only avoids the possible toxic and side effects of drugs but also solves the patients' doubts that the use of a large number of drugs may have an impact on fetal health in the future; ② two-way regulation can kill many birds with one stone. Pelvic floor muscle massage can regulate the balance of yin and yang, regulate the profit and loss of qi and blood of Zang Fu organs, strengthen the function of Zang Fu organs, and improve the ovarian uterine blood perfusion during embryo implantation, so as to improve the pregnancy rate; and ③ Simple operation and low cost. In this study, ssa-600e massager of Shanghai Shengsheng medical instrument company is used, which has no trauma and pain, good patient compliance, simple operation, low-cost, and no economic burden. The pelvic floor muscle belongs to the perineum muscle, which is a group of pelvic diaphragm and urogenital diaphragm separating the small pelvic cavity and perineum. It is composed of three layers of muscles and fascia to close the pelvic outlet. There is a pelvic diaphragm fissure in the front of the pelvic diaphragm. The urogenital diaphragm strengthens the pelvic floor from below, with urethra and vagina passing through. The pelvic diaphragm is located in the anal triangle, with rectum passing through, supporting and maintaining the pelvic organs in the normal position. It can control urination, maintain vaginal contraction, and enhance pleasure and other physiological functions. Under normal circumstances, pelvic floor muscle contraction is mostly caused by orgasm. For many infertile patients, it is difficult to reach orgasm and even have difficulty in sexual life, which is difficult to cause pelvic floor muscle contraction. Therefore, pelvic floor muscle cannot be exercised for a long time, its contractility is poor, and it cannot be congested, resulting in ischemia of various pelvic organs and insufficient nutrition. Patients with secondary infertility suffer from excessive pressure on pelvic floor muscles, muscle fiber deformation, decreased muscle tension, and pelvic muscle relaxation due to previous pregnancy, resulting in dissatisfaction with sexual life, stress urinary incontinence, uterine prolapse, incomplete closure of internal sphincter, and so on. Pelvic floor muscle weakness syndrome and pelvic congestion syndrome can lead to reduced uterine blood filling, endometrial dysplasia, difficult embryo implantation, and an increase in infertility patients. Therefore, the use of pelvic floor muscle massage can significantly improve the function of pelvic floor muscle through the massage effect of pelvic floor muscle, so as to improve the development of endometrium and improve the clinical pregnancy rate.

RETRACTED

All kinds of literatures show that the application of traditional Chinese medicine in IVF-ET has made a beneficial attempt. The research shows that the role of traditional Chinese medicine in regulating endometrial receptivity is positive. In assisted reproductive technology, the application of various traditional Chinese medicine means to improve the pregnancy rate reflects the idea of “prevention before disease” in traditional Chinese medicine. Zhang and others conducted a series of studies on the use of kidney tonifying traditional Chinese medicine to promote angiogenesis. On this basis, they put forward the theory of “tonifying the kidney and generating blood vessels,” which enriched the theoretical connotation of “kidney governing reproduction” and further revealed the essence of kidney tonifying theory. Traditional Chinese medicine uses the prescriptions of tonifying the liver and kidney, supplementing qi, harmonizing blood and promoting blood circulation to improve the pregnancy rate of assisted reproductive technology, and mainly tonifying the kidney. In this study, combined with the shock method in traditional Chinese medicine massage, the simple use of physical therapy enables many patients who are unwilling to take traditional Chinese medicine or have concerns about drugs to better cooperate with the treatment. Through the combination of massage and acupoint massage, the overall adjustment is carried out in multiple ways, multiple levels, and multiple targets, so as to combine the syndrome differentiation and treatment of traditional Chinese medicine with the pregnancy assistance technology of Western medicine, develop their strengths, and avoid their weaknesses. It opens up a new way to improve the success rate of assisted reproductive technology. With the development of in vitro fertilization embryo transfer technology, laboratory technology is becoming more and more perfect, because the impact of technical reasons on embryos is becoming smaller and smaller. The main factors affecting the success rate of IVF-ET focus on the patient's own embryo quality, endometrial receptivity (ER) ,and so on. Pelvic floor muscle massage can improve endometrial receptivity. Endometrial receptivity refers to the ability of endometrium to accept embryos [17]. In the normal reproductive cycle of human and mammals, there is only a very short period of endometrium that allows embryo implantation. This period is called “implantation window period,” at which the endometrium shows the greatest receptivity. If embryonic development is not synchronized with endometrial receptive development, or poor receptivity is not suitable for embryo implantation, it will lead to pregnancy failure. At present, the research on endometrial receptivity mainly focuses on pinopodes, subendometrial blood flow, integrins, leukemia inhibitory factor (LIF), etc. Pelvic floor muscle massage mainly affects the blood flow under the endometrium.

RETRACTED

In conclusion, this study found that pelvic floor muscle massage can effectively improve the clinical pregnancy rate. The mechanism is to induce muscle contraction, increase intra-abdominal pressure, accelerate pelvic blood flow, reduce the blood flow resistance of uterine artery, and increase the subendometrial blood flow and blood perfusion, so as to improve the thickness and structure of endometrium and improve the active function and hormone level of uterus and ovary. The improvement of the intrauterine environment, the development of pinocytes, the expression of integrin and leukemia inhibitory factor, and the increase of endometrial receptivity are conducive to embryo implantation.

## Figures and Tables

**Figure 1:** Classification criteria for subendometrial blood flow of each type.

**Figure 2:** Comparison of the intima and embryonic conditions of the patients in the two groups.

**Table 1:** Comparison of the intima and embryonic conditions of the patients in the two groups.

Index	Control group (*n* = 60)	Research group (*n* = 60)	Statistic value	*P* value
Inner al membrane thickness on the second day of menstruation	0.49 ± 0.03	0.45 ± 0.02	8.593	0.05
Flavestin anterior inner membrane thickness	1.17 ± 0.03	1.20 ± 0.04	-4.647	0.001
A-type intima	47	52	1.443	0.230
The number of excellent embryo	2.61 ± 0.15	2.89 ± 0.21	-8.404	0.001
Transplant number	1.85 ± 0.73	2.02 ± 0.24	-1.713	0.089

**Table 2:** Comparison of subendometrial blood flow type and blood flow index in the two groups.

Index	Control group (*n* = 60)	Research group (*n* = 60)	Statistic value	*P* value
Menstrual 10 d			0.137	0.711
III + II	36	34		
I	24	26		
Menstrual 17 d			1.725	0.001
III + II	37	56		
I	23	4		

**Table 3:** Comparison of pregnancy outcomes between the two patient groups.

Index	Control group (*n* = 60)	Research group (*n* = 60)	Statistic value	*P* value
Biochemical pregnancy	38	24	6.541	0.011
Clinical pregnancy	26	36	3.337	0.068
Early abortion	2	1	0.342	0.559
Eccyesis	1	0	0.135	0.843

## Data Availability

The data used to support this study are available from the corresponding author upon request.
